# The Impact of Seeding Density and Nitrogen Rates on Forage Yield and Quality of *Avena sativa* L

This article has been retracted.

**DOI:** 10.1155/2022/8238634

**Published:** 2022-06-30

**Authors:** Aroosa Kanwal, Dawood Zubair, Rao Mehboob ur Rehman, Muhammad Ibrahim, Muhammad Amjad Bashir, Muhammad Mudassar Maqbool, Muhammad Imran, Ubaid ur Rehman, Omaima Nasif, Mohammad Javed Ansari

**Affiliations:** ^1^Rural Health Center, Bhekho More District, Mandi Bahauddin, Punjab, Pakistan; ^2^ER Medical Officer at Iqra Medical Complex, Johar Town Lahore, Pakistan; ^3^Hamdard College of Medicine and Dentistry, Hamdard University, Karachi, Pakistan; ^4^Department of Agronomy Faculty of Agricultural Sciences, Ghazi University, Dera Ghazi Khan Punjab, Pakistan; ^5^Department of Plant Protection Faculty of Agricultural Sciences, Ghazi University, Dera Ghazi Khan Punjab, Pakistan; ^6^Department of Soil and Environmental Sciences, MNS University of Agriculture, Multan Punjab, Pakistan; ^7^United States Department of Agriculture, Washington DC, USA; ^8^Department of Physiology, College of Medicine, King Khalid University Hospital, King Saud University, Medical City, PO Box 2925, Riyadh 11461, Saudi Arabia; ^9^Department of Botany, Hindu College Moradabad (Mahatma Jyotiba Phule Rohilkhand University Bareilly), India

## Abstract

Green forage is an excellent feed source for livestock. It is an integral part of livestock production to accomplish the demands for butter, milk, and other derivatives for human utilization. Livestock contributes 11.39% towards the gross domestic product of Pakistan and 58.33% in agricultural farming. Livestock face shortage or insufficient supply of green fodder during the winter season, which ultimately reduces milk yield. Oat (*Avena sativa* L.) is a major forage crop in the winter season; however, several biotic and abiotic factors negatively affect its yields. Low soil fertility, particularly nitrogen deficiency, is regarded as one of the few reasons responsible for the low forage yield of oat. Low organic matter content in the soil, suboptimal agronomic practices, and harsh climatic conditions are the other major reasons for low oat yield. Seed rate and different nitrogen rates significantly alter green forage yield and quality of oat. This study assessed the impact of different seeding densities and nitrogen (N) doses on the forage yield of oat. Three seeding densities (70, 80, and 90 kg ha^−1^) and five N doses (0, 40, 80, 120, and 160 kg ha^−1^) were included in the study. The interactive effect of seeding density and N doses significantly altered green forage yield and quality attributes of oat. The highest green forage yield (54.67 t ha^−1^) was noted for the interaction among 90 kg seed rate ha^−1^ and 160 kg N ha^−1^. Similarly, the highest germination count (140 m^−2^), number of tillers (5.97 m^−2^), plant height (122.97 cm), number of leaves per plant (24.50 m^−2^), leaf area per tiller (123.18 cm^2^), fresh weight (5.47 kg m^−2^), dry weight (1692 g m^−2^), dry matter yield (20.90 t ha^−1^), crude protein (10.54%), crude fiber (31.62%), and total ash (9.39%) were recorded for the interactive effect of 90 kg seed rate ha^−1^ and 160 kg N ha^−1^. Economic analysis revealed that interaction between 90 kg seed rate ha^−1^ with 120 and 160 kg N ha^−1^ was superior to others with higher benefit: cost ratio and net economic returns. It is recommended that the oat seed rate of forage oat crop must be kept at 90 kg ha^−1^ and it should be supplied 120 kg N ha^−1^ for higher yield, better quality, and more economic returns.

## 1. Introduction

Green forage is a valuable and the cheapest source of energy and provides excellent feed for livestock. A sustainable supply of green forage is a major constraint in livestock production to achieve the requirements for milk, butter, and other milk derivatives for human consumption [1]. Livestock contributes 58.33% towards agriculture and 11.39% towards the gross domestic product of Pakistan during 2016-2017 [2]. Livestock is usually underfed in Pakistan, which results in a low animal population. Imbalanced and low soil fertility, low organic matter content, and nitrogen deficiency are the major factors responsible for the low forage yield globally [3].

Oat is locally known as “jai” or “jodar” in Pakistan and belongs to the family Poaceae. Pakistan is facing a 52-54% deficiency in the domestic fodder requirements [4]. Globally, oat is grown for grain, green forage, and fodder for livestock. It is the most important and cheapest source of cereal fodder crops grown during the winter season throughout Pakistan under rain-fed and irrigated conditions. Oat fodder is nutritious, palatable, and succulent. The nutritive value of oat fodder can be increased by combining it with legumes, like alfalfa, Persian clover, berseem, and pea [5]. It contains high amounts of minerals, including phosphorus and iron, fat, vitamin B_1_, and protein. Oat is a high-yielding crop in temperate climates and exhibits low tolerance to waterlogging [1]. Oat grains are a rich nutritive feed for dairy cows, sheep, horses, and young breeding animals [6]. Oat forage contains 30.44% crude fiber, 9.3% crude protein, 3.56% fat, and 0.27% phosphorus. It can be directly grazed to feed animals before seed setting and can be grown for grain purposes [7]. Its good quality grains and leaves are a rich source of carotene and carbohydrates. Oat requires 16-32°C temperature and 400 mm rainfall during the growing season for optimum growth and development [8].

Grains and leaves of forage oat are a rich source of carotene and carbohydrates [7]. The forage yield of oat in Pakistan is too low than other countries. The main reasons for low forage production are changing climate, low soil fertility, unavailability of high-yielding varieties, socioeconomic factors, shortage of irrigation water, poor seeding techniques, and mismanagement of fertilizer application [9].

Genus *Avena* consists of seventy species. *Avena byzantina* and *Avena sativa* are mainly cultivated for green forage and fodder purposes. There is a dire need to improve the forage yield of oat, which can be achieved by adopting improved agronomic practices [8]. Oat ranks 6^th^ as a cereal crop worldwide after wheat, maize, rice, barley, and sorghum. Oat is a multicut fodder crop and achieves maximum green fodder yield with appropriate management. It should be harvested at 50% flower blooming [10].

Sowing fodder crops with optimum seed rate is important to get sufficient plant population, which ultimately contributes towards high forage production. Plant population has a direct impact on forage yield and quality. Low and high plant population reduces the yield and quality of forages; thus, seeding density must be kept optimum. The seed rate of legumes could be decreased when these are sown in a mixture with other fodders [11, 12] The use of low or high seed rate exerts negative impacts on forage yield and quality [13]. A lower seed rate increases plant height, while a high seed rate reduces plant height due to less space, antagonism for light, and other resources [14]. The plant height of forage crops decreases with increasing seeding rate, which indicates competition for light [14].

Kakol et al. [15] recorded the highest green forage yield of oat with a 100 kg ha^−1^ seed rate compared to 125 kg ha^−1^, while the quality of forage remained unaffected. Jan and Jan [16] have also reported a nonsignificant impact of seed rates on green and dry forage yields of oat. Abate and Wegi [13] concluded that optimum seed rate and fertilizer level have a significant effect on green forage yield of oat and dry matter production.

Nitrogen (N) is a compulsory part of protein and a physiologically important compound that improves the growth and development of crop plants [17]. Nitrogen plays a vital role in crop production [18–20]. It is an essential ingredient of plant cell constituents like green pigments, amino acids, enzymes, and nucleic acids. Plants uptake N in dissolved form and partition it into different organs. Nitrogen exerts significant impacts on tillering, stem elongation, heading, cell division, booting, and grain filling. Nitrogen also affects crop morphology [21]. It is the most deficient nutrient in soils, thus required in heavy amounts for cereal and fodder crops [22]. Several factors including soil pH, moisture contents, and temperature significantly affect N losses [23]. However, the application of optimum dose is important to fetch high yield and quality [16]. Higher N application improves forage yield. Green fodder yield of oat was significantly affected by 80 kg N ha^−1^, and it was higher than control, 40 and 120 kg ha^−1^ [24]. However, the optimum N dose significantly varies among locations and agroclimatic conditions. Therefore, it is mandatory to optimize the N application dose and seed rate for high forage production. It was hypothesized that increasing the N dose will significantly differ the forage yield and quality. Similarly, different seed rates would have a significant impact on forage yield and quality of oat. The results will help to optimize seed rate and N doses for oat fodder production in agroclimatic conditions of Dera Ghazi Khan, Pakistan.

## 2. Materials and Methods

### 2.1. Experimental Site

The current field study to optimize seed rate and N application rate for oat were conducted at a research farm, Ghazi University, Dera Ghazi Khan, Pakistan, during the winter season, 2015-2016.

### 2.2. Experimental Details

The experiment was conducted on a fallow field, which was leveled, and fallow cultivation was done. Thereafter, presocking irrigation of 10 cm was applied, and the field was cultivated two times with the help of a cultivator followed by planking when the soil attained a workable moisture regime. The approved oat cultivar for forage production (S-2000) was used in the experiment. Three seed rates, i.e., 70, 80, and 90 kg ha^−1^, and five N levels (0, 40, 80, 120, and 160 kg ha^−1^) were included in the study. Seeds were sown in 30 cm-apart rows with the help of a single-row hand drill, and each experimental unit consisted of six lines. The crop was sown during the 2^nd^ week of December 2015. Urea and single super phosphate (SSP) were used as the source of nitrogen and phosphorus, respectively. The whole amount of recommended phosphorus rate (80 kg ha^−1^) was applied as a basal dose, while N was applied in two splits according to the treatments. The first split of N was applied at the time of sowing, whereas the second split was given with the first irrigation. Three irrigations were given during the entire growth period of the crop. The crop was harvested manually at a ground level with the help of a sickle date.

### 2.3. Data Collection

Standard procedures were used for data collection which were kept uniform for all treatments. Data relating to germination count (m^−2^), plant height (cm), number of leaves (per plant), number of tillers (m^−2^), leaf area per tiller (cm^2^), fresh weight (kg m^−2^), dry weight (g m^−2^), green forage yield (t ha^−1^), and dry matter yield (t ha^−1^) were collected. For seed germination, experimental plots were visited daily until the last seed emerged. The number of seeds germinated on the final day of the count was regarded as germination count. The heights of five randomly selected plants from each experimental unit were measured and averaged. The number of tillers from five randomly selected plants in each experimental unit was counted and averaged. The destructive sampling method was used for the determination of fresh and dry biomass. A 1 m^2^ area was harvested and weighed to record fresh forage yield. The harvested sample was dried in an oven at 70°C, and then the dry yield was measured. This yield was then converted to t ha^−1^ by a unitary method. Crude protein (%), crude fiber (%), and total ash (%) were determined by burning a predefined quantity of the plants.

### 2.4. Economic Analysis

Economics analysis was conducted to determine the economic feasibility of applied treatments. Total and gross incomes were calculated from the total yield of the forage oat. Then the total cost of production was calculated by adding total fixed and total variable costs. Benefit-cost was determined by dividing the gross income by the total cost according to the procedures devised by CIMMYT (1988).

(1) $$\begin{array}{c} \text{Benefit}-\text{cost ratio}=\frac{\text{Net income}}{\text{Total expenditure}}. \end{array}$$

### 2.5. Statistical Analysis

The collected data of all parameters were analyzed by Fisher‘s analysis of the variance technique, and the LSD test at a 0.05 probability level was applied to compare the significance of treatment means [25].

## 3. Results

### 3.1. Germination Count (m^−2^)

The germination count of forage oat was significantly affected by different seed rates, while the main effects of the N level were nonsignificant (Table 1). Similarly, the interactive effect of the seed rate and N level was also nonsignificant. The highest germination count was recorded for S_3_ (138.77 m^−2^), whereas the lowest plant population (108.42 m^−2^) was noted for S_1_ (Table 2). The higher germination count is directly linked to a higher seed rate used.

### 3.2. Morphological Attributes

The individual and interactive effects of seed rate and N doses significantly altered plant height, number of leaves per plant, leaf area per tiller, and fresh and dry weight (Table 1). The highest plants were observed for S_2_N_5_ (122.97 cm), which was statistically at par with S_1_N_5_, S_3_N_5_, S_3_N_4_, and S_1_N_4_. The lowest plant height was observed for S_2_N_1_ (91.37 cm), S_1_N_2_ (94.37 cm), S_1_N_1_ (94.43 cm), and S_1_N_3_ (96.33 cm). The increase in N unit increased plant height (Table 2).

More number of leaves of forage oat were noted for S_3_N_5_ (24.50 m^−2^), which was statistically similar to S_2_N_5_, S_3_N_4_, and S_2_N_4_. The lowest numbers of leaves per plant were recorded for S_2_N_1_, which was statistically similar to S_1_N_1_, S_1_N_2_, and S_3_N_1_ (Table 2).

The highest leaf area was recorded for S_2_N_5_, which was statistically similar to S_3_N4, S_1_N_5_, S_3_N_2_, and S_3_N_5_. The lowest leaf area was observed for S_1_N_1_, and it was closely related to S_1_N_2_ and S_1_N_3_ (Table 2).

### 3.3. Yield and Quality Attributes

The individual and interactive effects of seed rate and N doses significantly affected forage yield, dry matter yield, crude fiber, crude protein, and total ash in forage oat (Table 3). Overall, these parameters were increased with increasing seed rate and N levels. The highest green forage yield was noted for S_3_N_5_, which was similar to S_3_N_4_, S_2_N_5_, and S_2_N_4_ (Table 4). The lowest green forage yield was produced by S_1_N_1_, and it was statistically similar to S_2_N_1_ and S_3_N_1_. Kakol et al. (2003) reported that oat plants positively respond to seed rate and N, which improve their growth and forage production. Shukla and Lal (1998) recorded significant differences among 80 and 60 kg phosphors for green forage yield. The highest dry matter yield was observed for S_1_N_4_, whereas S_1_N_1_ recorded the lowest dry matter yield (Table 4).

Variation in seed rate and N level significantly affected the crude fiber percentage. The highest crude fiber percentage was observed for S_3_N_5_, while S_2_N_1_ resulted in the lowest crude fiber percentage (Table 4).

### 3.4. Economic Analysis

The interactive effect of seed rate and N doses has a significant impact on variable costs (Table 5) and economics (Table 6). The highest net income and benefit-cost ratio was recorded for S_3_N_4_, whereas S_1_N_1_ recorded the lowest net income and benefit-cost ratio, although increasing N doses improved all traits and the highest dose proved superior in this regard. However, the economic analysis revealed that applying higher N doses is not an economic option. Although the highest N dose, i.e., N_5_, also recorded a higher net income and benefit-cost ratio than other N doses, N_4_ recorded the highest net income and benefit-cost ratio (Table 6).

## 4. Discussion

The higher germination count is directly linked to a higher seed rate used. These results are similar to [26] who recorded the highest number of plants of forage maize with a higher seeding density. The nonsignificant effect of N doses on germination of forage oat is also reported by Shukla and Lal [27] who also reported nonsignificant results of oat germination percentage when grown with organic or inorganic sources of fertilizers. This might be due to the contribution of N in the growth of oat plants. Zahid et al. [28] concluded that plant height was increased with increasing N doses and farmyard manure. Irfan et al. [29] found a significant difference in the plant height of oat, and these results are also in line with others. Another concluded that the plant height of oat was significantly altered by the split application of N and potassium. One of them recorded significantly higher plant height (119.58 cm) in forage oat by the application of 80 kg N ha^−1^.

The higher number of leaves per plant can be owed to the contribution of N in vegetative growth. Similar findings have been reported by Ahmad et al. [30]. Irfan et al. [29] reported higher and lower numbers of leaves of forage oat with the highest and the lowest N application.

The highest number of tillers m^−2^ was counted for S_3_N_5_, which was similar to S_3_N_4_, S_2_N_5_, S_3_N_3_, and S_3_N_2_. The lowest number of tillers per plant in forage oat was observed for S_1_N_1_, which was statistically similar to S_2_N_1_, S_3_N_1_, and S_1_N_2_ (Table 2). Metwally et al. [31] concluded that the application of 100 kg ha^−1^ N significantly enhanced the tillering capacity of forage oat. Jehangir et al. [32] reported that the number of tillers significantly increased with increasing the fertility status of the soil. These results are in line with Ahmad et al. [30] who concluded that 150 kg ha^−1^ N and 60 kg ha^−1^ phosphorus produces the highest leaf area of (128 cm^2^) in forage oat. Jiwang et al. [33] reported that increasing the fertilizer level increases the leaf area. Khandaker and Islam [34] recorded the highest leaf area of forage oat with 120 kg ha^−1^ N. Tanha [35] observed the highest leaf area in forage maize with 200 kg ha^−1^ N application.

Fresh and dry weights significantly increased with the increasing seed rate and N level. The highest fresh weight was observed for S_3_N_5_, which was close to S_3_N_4_. The lowest fresh weight was observed for S_1_N_1_. Sharma and Bhunia [36] studied the response of organic and inorganic sources of N and concluded that the inorganic N source produced the highest fresh weight per tiller. Singh et al. [37] reported that the application of farmyard manure significantly increased the fodder yield in maize. Wheed et al. [38] reported that a higher N level increased green forage yield.

Orloff et al. [39] recorded the highest dry fodder yield with 136 kg ha^−1^ N application.

Crude protein percentage is an important quality parameter, which determined the quality of forage crops. Application of N from lower to higher levels significantly increased crude protein contents; however, crude protein beyond a certain range reduced the forage quality and increases succulence. The highest crude protein was observed for S_2_N_5_, whereas S_2_N_1_ resulted in the lowest crude protein. Kumar et al. [40] observed that 80 kg ha^−1^ N resulted in the maximum crude protein yield and observed a maximum crude protein yield with 120 kg N ha^−1^. Kumar et al. [41] observed that the application of N up to 80 kg per hectare enhanced the crude protein yield, and a further increase in N decreased the crude protein yield. Khan et al. [42] concluded that crude protein quality may be affected by N application as it is an essential part of protein, chlorophyll, and protoplast. Farooq et al. [43] also reported similar results. These results are in line with [44] who observed higher crude fiber with 150 kg ha^−1^ N application.

The highest ash percentage was recorded for S_3_N_4_, and the lowest was observed for S_1_N_1_ (Table 4). These results are in line with Alajmi et al. [45] who observed a maximum ash percentage with 150 kg ha^−1^ N application. Saleh et al. [46] also concluded similar results and reported that increasing N application significantly increased the ash content in forage maize.

## 5. Conclusion

The results revealed that seed rate and nitrogen doses significantly altered the yield and forage quality of forage oat. It is concluded that forage oat crops should be grown with a seed rate of 90 kg ha^−1^ and supplemented with 120 kg ha^−1^ of nitrogen for higher yield, better quality, and more economic returns.

## Figures and Tables

**Table 1:** Analysis of variance of different seeding rates, nitrogen doses, and their interactions on germination count, plant height, number of tillers per plant, leaf area per tiller, and fresh and dry biomass of oat.

SOV	DF	SS	MS	*P* value
*Germination count*				
Seed rate (S)	2	6932.5	3466.25	0.0000^∗∗^
Nitrogen doses (N)	4	994.2	248.56	0.0852NS
S × N	8	1168.6	146.08	0.2640NS
*Plant height*				
Seed rate (S)	2	359.69	179.85	0.0028^∗^
Nitrogen doses (N)	4	4829.57	1207.39	0.000^∗∗^
S × N	8	569.46	71.18	0.0173^∗^
*Number of tillers*				
Seed rate (S)	2	9.9613	4.98067	0.0000^∗∗^
Nitrogen doses (N)	4	25.3444	6.33611	0.0000^∗∗^
S × N	8	2.5542	0.31928	0.00136^∗^
*Leaf area per tiller*				
Seed rate (S)	2	1570.23	785.114	0.0000^∗∗^
Nitrogen doses (N)	4	2863.32	715.831	0.0000^∗∗^
S × N	8	883.81	110.476	0.0235^∗^
*Fresh weight*				
Seed rate (S)	2	3.4964	1.74822	0.0000^∗^
Nitrogen doses (N)	4	32.3658	8.09144	0.0000^∗∗^
S × N	8	0.1969	0.02461	0.0240^∗^
*Dry weight*				
Seed rate (S)	2	287097	143548	0.0008^∗^
Nitrogen doses (N)	4	7122222	1780555	0.0000^∗∗^
S × N	8	534114	66764	0.0016^∗^

SOV: source of variation, DF: degree of freedom, SS: sum of squares, MS: mean squares, ^∗^: significant, NS: nonsignificant.

**Table 2:** Interactive effect of seed rate and nitrogen level on germination count, plant height, numbers of leaves, and leaf area per tiller of forage oat.

Treatments	Germination count (m^−2^)	Plant height (cm)	Number of leaves (m^−2^)	Leaf area per tiller (cm^2^)	Fresh weight (kg m^−2^)	Dry weight (g m^−2^)
*Seed rate (S)*						
S_1_	108.42 C	104.45 B	20.180 B	110.08 B	3.8267 C	897.7 B
S_2_	125.19 B	108.1 AB	20.780 B	118.32 A	4.2200 B	845.3 B
S_3_	138.77 A	111.37 A	22.060 A	100.02 C	4.5067 A	1034.7 A
LSD	3.8	1.8	0.32	2.33	0.34	45.13
*Nitrogen doses (N)*						
N_1_	119.93 NS	92.51 D	19.667 D	107.00 B	2.7889 E	457.6 C
N_2_	118.64	103.48 C	17.756 E	117.81 A	3.7444 D	468.1 C
N_3_	123.08	105.32 C	20.956 C	121.95 A	4.3333 C	1008.9 B
N_4_	128.47	116.71 B	22.756 B	94.91 de	4.9556 B	1342.0 A
N_5_	130.61	121.90 A	23.900 A	96.54 de	5.1000 A	1353.0 A
LSD 0.05	4.91	2.33	0.42	90.54 e	0.44	58.26
*S* × *N*						
S_1_N_1_	109.97 NS	94.43 g	17.50 g	115.91 ab	2.47 k	403.0 e
S_1_N_2_	103.23	94.37 g	17.67 fg	121.61 a	3.23 h	459.7 e
S_1_N_3_	101.70	96.33 fg	20.63 d	102.15 cd	4.03 fg	962.7 cd
S_1_N_4_	115.97	115.70 abc	22.20 c	104.71 cd	4.63 d	1317.3 b
S_1_N_5_	111.23	121.40 ab	22.90 bc	104.58 cd	4.77 d	1346.0 b
S_2_N_1_	111.2	91.37 g	17.43 g	115.78 ab	2.87 j	494.0 e
S_2_N_2_	114.53	104.50 ef	19.10 ef	123.18 a	3.90 g	470.7 e
S_2_N_3_	129.13	106.30 de	20.03 de	107.38 bc	4.33 e	1167.3 bc
S_2_N_4_	131.23	115.57 abc	23.03 abc	121.54 a	4.93 c	1016.7 cd
S_2_N_5_	139.87	122.97 a	24.30 ab	119.88 a	5.07 c	1348.3 b
S_3_N_1_	138.33	91.73 g	18.33 fg	121.74 a	3.03 i	475.7 e
S_3_N_2_	138.17	111.57 cde	22.23 c	121.08 a	4.10 f	474.0 e
S_3_N_3_	138.4	113.33 bcd	22.20 c	10.65	4.63 d	896.7 d
S_3_N_4_	138.2	118.87 abc	23.03 abc	110.77	5.30 b	1692.0 a
S_3_N_5_	140.73	121.33 ab	24.50 a		5.47 a	1364.7 b
LSD 0.05	17.44	8.29	1.48		0.16	206.7
Mean	124.13	107.98	21		4.18	19.32

Here, S_1_ = 70 kg ha^−1^, S_2_ = 80 kg ha^−1^, S_3_ = 90 kg ha^−1^, N_1_ = 0 kg ha^−1^, N_2_ = 40 kg ha^−1^, N_3_ = 80 kg ha^−1^, N_4_ = 120 kg ha^−1^, and N_5_ = 160 kg ha^−1^. Means sharing similar letters within a column are statistically nonsignificant.

**Table 3:** Analysis of variance of different seeding rates, nitrogen doses, and their interactions on forage and dry matter yields, crude fiber, crude protein, and total ash of forage oat.

SOV	DF	SS	MS	*P* value
*Forage yield*				
Seed rate (S)	2	338.71	169.356	0.0000^∗∗^
Nitrogen doses (N)	4	3213.35	803.338	0.0000^∗∗^
S × N	8	28.89	3.612	0.0151^∗^
*Dry matter yield*				
Seed rate (S)	2	3.7773	1.8887	0.0008^∗^
Nitrogen doses (N)	4	83.3142	20.8286	0.0000^∗∗^
S × N	8	4.2604	0.5326	0.0268^∗^
*Crude protein*				
Seed rate (S)	2	1.2379	0.6189	0.0304^∗^
Nitrogen doses (N)	4	72.2770	18.0692	0.0000^∗∗^
S × N	8	6.8236	0.8529	0.0003^∗^
*Crude fiber*				
Seed rate (S)	2	53.324	26.6618	0.0037^∗^
Nitrogen doses (N)	4	226.558	56.6395	0.0000^∗∗^
S × N	8	97.847	12.2309	0.0111^∗^
*Total ash*				
Seed rate (S)	2	9.3352	4.66760	0.0000^∗∗^
Nitrogen doses (N)	4	11.2192	2.80480	0.0000^∗∗^
S × N	8	4.8808	0.61010	0.0029^∗^

SOV: source of variation, DF: degree of freedom, SS: sum of squares, MS: mean squares, ^∗^: significant, NS: nonsignificant.

**Table 4:** Interactive effect of seed rate and nitrogen level on green forage yield, dry matter yield, crude protein, crude fiber, and total ash of forage oat.

Treatments	Green forage yield (t ha^−1^)	Dry matter yield (t ha^−1^)	Crude protein (%)	Crude fiber (%)	Total ash (%)
*Seed rate (S)*					
S_1_	38.827 C	19.07 B	8.87 A	27.28 B	7.58 C
S_2_	42.717 B	19.16 B	8.52 A	27.10 B	7.91 B
S_3_	45.517 A	19.73 A	8.88 B	29.49 A	8.67 A
LSD 0.05	0.4	0.16	0.14	0.72	0.14
*Nitrogen doses (N)*					
N_1_	28.389 E	17.17 D	6.98 E	24.75 C	7.14 C
N_2_	37.978 D	18.57 C	7.82 D	26.76 B	7.93 B
N_3_	43.983 C	19.40 B	8.72 C	27.36 B	8.30 AB
N_4_	50.170 B	20.64 A	9.86 B	29.88 A	8.44 A
N_5_	51.249 A	20.87 A	10.42 A	31.03 A	8.48 A
LSD 0.05	0.51	0.21	0.19	0.92	0.18
*S* × *N*					
S_1_N_1_	25.833 i	16.60 d	7.45 ef	24.55 d	6.57 e
S_1_N_2_	32.600 g	18.07 c	8.23 d	24.71d	7.02 e
S_1_N_3_	41.033 ef	19.33 b	8.41 d	27.75 bcd	8.00 cd
S_1_N_4_	46.667 c	20.57 a	9.80 bc	29.32 abc	7.88 cd
S_1_N_5_	48.000 c	20.80 a	10.45 ab	30.05 ab	8.45 bc
S_2_N_1_	29.000 h	16.70 d	5.94 g	20.55 e	6.78 e
S_2_N_2_	39.667 f	18.23 c	7.22 f	26.22 cd	7.79 d
S_2_N_3_	43.917 d	19.43 b	9.27 c	27.15 bcd	8.45 bc
S_2_N_4_	49.923 b	20.63 a	9.93 abc	30.15 ab	8.05 cd
S_2_N_5_	51.080 b	20.80 a	10.28 ab	31.42 a	8.49 bc
S_3_N_1_	30.333 h	18.20 c	7.54 ef	29.15 abc	8.05 cd
S_3_N_2_	41.667 e	19.37 b	8.00 de	29.35 abc	8.99 ab
S_3_N_3_	47.000 c	19.43 b	8.49 d	27.18 bcd	8.45 bc
S_3_N_4_	53.920 a	20.90 a	9.85 bc	30.15 ab	9.39 a
S_3_N_5_	54.667 a	20.73 a	10.54 a	31.62 a	8.49 bc
LSD 0.05	1.84	0.75	0.66	3.29	0.65
Mean	42.35	19.32	8.76	27.95	8.06

Here, S_1_ = 70 kg ha^−1^, S_2_ = 80 kg ha^−1^, S_3_ = 90 kg ha^−1^, N_1_ = 0 kg ha^−1^, N_2_ = 40 kg ha^−1^, N_3_ = 80 kg ha^−1^, N_4_ = 120 kg ha^−1^, and N_5_ = 160 kg ha^−1^. Means sharing similar letters within a column are statistically nonsignificant.

**Table 5:** Fixed and variable costs of production for forage oat.

Operation/input	No. of operations/ha	Rate per unit (PKR)	Cost per unit (PKR)
*Land preparation*			
Ploughing	2	2000 ha^−1^	4000 ha^−1^
Planking	1	1500 ha^−1^	1500 ha^−1^
*Sowing*			
Seed/sowing	^∗^	^∗^	^∗^
Drill sowing		2500 ha^−1^	2500 ha^−1^
*Irrigation*			
Irrigation charges	3 irrigations	1000	3000
Labor cost for irrigation	1 man for 3 times	500 per day	1500
*Fertilizer*			
Nitrogen from urea	^∗^	^∗^	^∗^
Phosphorus from single super phosphate	80 kg	111 kg^−1^	8888
Plant protection measures	Weeding		1000
*Harvesting*			
Labor charges for harvesting	7 men	500 per men	3500
Land rent	6 months	30250 ha^−1^	15125
Total fixed cost			41013

^∗^: variable cost of seed, ^∗^: variable cost of nitrogen.

**Table 6:** Economics analysis for different seed rates and nitrogen doses used to produce forage oat.

Treatments	Gross income (PKR ha^−1^)	Total cost (PKR ha^−1^)	Net income (PKR ha^−1^)	Benefit : cost ratio
S_1_N_1_	51666	45213	6453	1.14
S_1_N_2_	65200	48253	16947	1.35
S_1_N_3_	82066	51293	30773	1.60
S_1_N_4_	93334	54333	39001	1.72
S_1_N_5_	96000	57373	38627	1.67
S_2_N_1_	58000	45813	12187	1.27
S_2_N_2_	79334	48853	30481	1.62
S_2_N_3_	87834	51893	35941	1.69
S_2_N_4_	99846	54933	44913	1.82
S_2_N_5_	102160	57973	44187	1.76
S_3_N_1_	60666	46413	14253	1.31
S_3_N_2_	83334	49453	33881	1.69
S_3_N_3_	94000	52493	41507	1.79
S_3_N_4_	107840	55533	52307	1.94
S_3_N_5_	109334	58573	50761	1.87

1 USD = 160 PKR. Here, S_1_ = 70 kg ha^−1^, S_2_ = 80 kg ha^−1^, S_3_ = 90 kg ha^−1^, N_1_ = 0 kg ha^−1^, N_2_ = 40 kg ha^−1^, N_3_ = 80 kg ha^−1^, N_4_ = 120 kg ha^−1^, and N_5_ = 160 kg ha^−1^.

## Data Availability

All data is available in the manuscript.
